# Study on Circulating lncRNA Expression Profile in Patients with Cerebral Infarction

This article has been retracted.

**DOI:** 10.1155/2022/3042105

**Published:** 2022-05-09

**Authors:** Man-tang Li, Cheng-hong Luo, Peng-jie Xu, Ya Jin

**Affiliations:** Department of Neurology, SSL Central Hospital of Dongguan City, Dongguan Third People's Hospital, Dongguan, 523320 Guangdong Province, China

## Abstract

To analyze the difference of circulating lncRNA expression profile between the healthy control group and cerebral infarction (CI) patients and to study the epigenetic pathogenesis of CI. Forty patients with acute CI admitted to our hospital from December 2016 to December 2017 were selected as CI group, and 40 healthy people in physical examination center were selected as healthy group. In the CI group, blood samples were taken 5 mL at fasting in the morning (within 72 hours of CI), and the blood samples from healthy group were also taken 5 mL at fasting in the morning. The circulating lncRNA expression profile of serum sample was determined by high-throughput technique, and its difference was analyzed. Bioinformatics technology was used to explore its functional mechanism, and GO, KEGG analysis, and gene expression network were established for lncRNA with significant differences. Next, lnc-ZNF32-1 : 1 and lnc-PCGF5-2 : 1 were selected for further validation of serum lncRNA expression in ACI and NC groups, and ceRNA interaction network analysis, diagnostic specificity, and sensitivity of lnc-ZNF32-1 : 1 and lnc-PCGF5-2 : 1 were conducted. The results showed that compared with the healthy group, there were 512 known lncRNA expressed differentially in the serum of patients with CI, of which 371 were upregulated and 141 were downregulated, and 421 known mRNA expressed differentially, of which 245 were upregulated and 176 downregulated. The differentially expressed mRNA was mainly enriched in 53 gene functions, and the target gene was enriched in the pathways such as HTLV-I infection and pathways in cancer. In addition, the results explored that lnc-ZNF32-1 : 1 and lnc-PCGF5-2 : 1 have potential value for CI diagnosis. In conclusion, the expression profile of lncRNA in CI group was significantly different from that in healthy group, indicating that lncRNA might be closely related to the occurrence, development, and prognosis of CI.

## 1. Introduction

Cerebral infarction (CI) is a general term for ischemic stroke. It is a brain lesion caused by cerebral blood supply disorders, including cerebral thrombosis, lacunar infarction, and cerebral embolism, which accounts for about 60-80% of cerebrovascular disease. There are 210-600 out of 100,000 people suffering from the disease each year, and about 20% of the deaths occur one month after the first onset [1–3]. CI is one of the most common cerebrovascular diseases in the clinic. It is the main cause of adult-acquired disability and the second leading cause of dementia. It has the characteristics of acute progression, rapid deterioration, and sudden onset. Patients with neurological dysfunction often accompanied by serious complications such as cerebral edema, cerebral palsy, myocardial infarction, and atherosclerotic CI [4–7]. At present, the treatment of CI is scarce, and only thrombolytic therapy in the window of 4.5 to 6 hours of onset is supported by evidence-based medical evidence [8]. Because of the high incidence of sequelae and the complicated pathologies of CI, medical researchers at home and abroad attach great importance to the study of its mechanism.

Long-chain noncoding RNA (lncRNA) is an RNA transcript of more than 200 nucleotides and plays an indispensable role in epigenetics [9, 10]. Recently, studies have found that lncRNA plays a genetic regulatory role in various biological processes such as cell growth, development, angiogenesis, and inflammatory response and is associated with many human diseases such as cancer, Alzheimer's disease, and cardiovascular disease [11–18]. The complexity of the mammalian brain is mainly due to the diversity of its neuronal and glial cell types. During brain development, the specification and differentiation of such cell types are spatially elaborated by the regulation of complex transcriptional programs. There is increasing evidence showing that lncRNA plays a key regulatory role in the process. In mammals, the largest lncRNA gene sequence and diversity occur in the brain and can exhibit regional and cellular specificity [19, 20]. The differential analysis of lncRNA expression profiles in patients with CI is rarely reported at home and abroad. In this study, we hypothesized that there are abnormal circulating lncRNA expression profiles of CI patients, and validation of these differences may provide new targets for the diagnosis or treatment of cerebral ischemia.

Therefore, the study mainly analyzed the differences in circulating lncRNA expression profiles between healthy controls and patients with CI and studied the epigenetic pathogenesis of CI, which provided a theoretical basis for finding new targets for the treatment of CI.

## 2. Material and Methods

### 2.1. Medical Records

Forty patients with acute CI admitted to our department of neurology from December 2016 to December 2017 were enrolled in the acute CI group (ACI group), and 40 healthy people were selected from the physical examination center as healthy control group (NC group). There were 40 patients in ACI group, 22 males and 18 females, aged 40-76 years, mean age (60.4 ± 23.4) years old; there were 40 patients in NC group, 20 males and 20 females, aged 42-74 years, mean age (61.8 ± 24.2) years. There was no significant difference in baseline characteristics between the two groups (*P* > 0.05). The study has been approved by the ethics committee of Dongguan Third People's Hospital, and informed signed consent was obtained from each participant.

### 2.2. Inclusion Criteria and Exclusion Criteria

Inclusion criteria: people confirmed by head CT or MRI, and in line with the diagnostic criteria for CI in Chinese CI Diagnosis and Treatment Guidelines by Integrated Chinese and Western Medicine (2017) [21]; acute onset; total focal neurological impairment or focal neurological impairment; nonvascular cause; hospitalization after 24 hours of the onset of CI; older than 40 years old; patient's family signed an informed consent form.

Exclusion criteria: unsatisfactory signs of illness, severe heart, kidney, liver, pulmonary insufficiency, failure or cancer; severe bleeding or coma; severe nervous or mental illness; cardiac CI caused by atrial fibrillation, arrhythmia, or rheumatic heart disease; major surgery within 4 weeks; patient or family disagree.

### 2.3. Methods

Specimen preparation: in the ACI group, blood samples were taken 5 mL at fasting in the morning after admission (within 72 hours of CI); blood samples from the healthy group were taken 5 mL in the morning on an empty stomach at the medical examination center. All samples were stored in a refrigerator at -80°C.

lncRNA sequencing: total RNA from the samples was extracted according to the instructions of Trizol kit (Invitrogen, USA). Then, ribosomal RNA was removed by rRNA probe hybridization digestion, and the product was randomly interrupted into RNA fragments. The RNA is then reverse transcribed into cDNA, and DNA concentration and purity were calculated by QPCR quantification using Agilent 2100 (Agilent Technologies, USA), followed by high-throughput sequencing on Illumina HiSeq TM 2000 (Illumina, USA). The obtained lncRNA and mRNA data were analyzed by DEseq for differentially expressed genes and the number of upregulated and downregulated genes.

Screening and cluster analysis of differentially expressed lncRNA and mRNA: after high-throughput sequencing with Illumina HiSeq TM 2000, followed by quality control of the raw reads to determine if the sequencing data is suitable for subsequent analysis, after quality control, filtered to obtain clean reads, and then the comparison software was used to compare the clean reads to the reference sequence. After the comparison, the distribution and coverage of the reads on the reference sequence are counted to determine whether the comparison result passes the second quality control. After quality control, a series of follow-up analyses are performed, such as gene expression, alternative splicing, new transcript prediction and annotation, and gene fusion. Differentially expressed lncRNA and mRNA in the two groups were represented by scatter plots, and hierarchical clustering analysis was performed.

GO, KEGC analysis of lncRNA target genes: the obtained *P* value is subjected to multiple hypothesis test correction, and the threshold of *P* value is determined by controlling FDR. In our analysis, differentially expressed genes were defined as genes with an FDR ≤ 0.001 and a fold difference of more than 2 fold. From the gene expression results, the differentially expressed genes between the samples were screened, and the GO significant functional enrichment analysis and pathway significant enrichment analysis were performed based on the differentially expressed genes.

GO analysis: GO analysis refers to the detection of functional properties of differentially expressed mRNA by analyzing differentially expressed mRNA data. GO has a total of three ontologies, which describe the molecular function, the cellular component, and the biological process of the genes. The degree of significance of the GO functional pathway was evaluated by the difference in the obtained *P* values, and the smaller the *P* value, the more significant the functional pathway.

KEGG analysis: KEGG is a database for analyzing gene function and genomic information and can analyze metabolic networks *in vivo*. Biological information analysis of differentially expressed mRNA was performed according to the KEGG database to analyze the biological pathways in which these differentially expressed mRNAs were mainly enriched. Then, the significance and false positive rate of the pathway were calculated, and the significance of the pathways these genes involved were screened out.

lncRNA gene expression network: the bioinformatics software was used to analyze the differentially expressed lncRNAs, and the genes in the most significant change trend models underwent coexpression network analysis to analyze which genes play a leading role in ACI. Based on the results of the lncRNA gene expression network, the diagnostic accuracy of ACI was evaluated, and the sensitivity, specificity, and accuracy of the diagnosis were analyzed.

### 2.4. qRT-PCR (Real-Time Quantitative Polymerase Chain Reaction)

Total RNA was extracted from blood samples with Trizol reagent (Invitrogen) and then processed with DNase I (Invitrogen) as directed. Oligo (dT) 20 and reverse transcriptase superscript II (Invitrogen) were employed to synthesize the first strand (cDNA). SYBR green PCR Master Mix (Qiagen, Hilden, Germany) was utilized to measure expressions of lnc-ZNF32-1 : 1 and lnc-PCGF5-2 : 1 using GAPDH as an endogenous control. A 2^-*ΔΔ*CT^ approach was used to analyze the data. Finally, the expression levels between groups were compared by unpaired *t*-test. *P* value < 0.05, means significant difference.

## 3. Results

### 3.1. Screening and Cluster Analysis of Differentially Expressed lncRNA in the Serum of ACI Group and NC Group

The lncRNA high-throughput sequencing technology was used to screen the differential expression of lncRNA in serum of ACI group and NC group. The results showed that there were 512 known differentially expressed lncRNAs, of which 371 were upregulated and 141 were downregulated. On this basis, the differentially expressed lncRNAs are clustered. Each column represents a sample. Each row represents a gene whose color indicates the amount of expression of the gene. The red represents upregulated genes, and blue represents downexpressed genes. The volcano plot and heat map are shown in Figures 1(a) and 1(b).

### 3.2. Screening and Cluster Analysis of Differentially Expressed mRNA in Serum of ACI Group and NC Group

High-throughput sequencing was used to screen for differential expressed mRNA in serum between ACI and NC groups. The results showed that there were 421 known differentially expressed mRNAs, of which 245 were upregulated and 176 were downregulated. Based on this, clustering analysis was performed on differentially expressed mRNAs. Each column represents a sample, and each row represents a gene. Its color indicates the amount of expression of the gene. The red represents upregulated genes, and blue represents downexpressed genes. The volcano plot and heat map are shown in Figures 2(a) and 2(b).

### 3.3. GO and KEGG Analysis of Differentially Expressed mRNA Gene in Serum of ACI Group and NC Group

As shown in Figure 3(a), GO analysis was performed on the differentially expressed genes of serum mRNA in ACI group and NC group, and the target genes with significant differences were selected for annotation (*P* < 0.05). These target genes are mainly enriched in 53 gene functions, which can be classified according to gene functions into 3 types: biological process, cellular components, and molecular function. It was found that differentially expressed mRNA is enriched in a number of biological processes associated with neurodevelopment and cardiovascular and cerebrovascular diseases.

The KEGG pathway analysis showed that the mRNA gene was mainly enriched in 6 pathways, and the target genes in the KEGG pathway database were enriched in HTLV-I infection, pathways in cancer, metabolism, MAPK, mTOR, PI3K-AKT, and other signaling pathways (Figure 3(b)). Many of these signaling pathways have been reported to be associated with ACI. The detailed results are shown in Table 1.

### 3.4. Verification of Differential Expression of lncRNA in ACI and NC Groups

To verify the differential expression of lncRNA in the sequencing results, we selected lnc-ZNF32-1 : 1 and lnc-PCGF5-2 : 1 for further qPCR detection in ACI group and NC group. The results of the validation showed that lnc-ZNF32-1 : 1 was significantly upregulated in the ACI group, consistent with the sequencing results; the expression of lnc-PCGF5-2 : 1 was downregulated in the ACI group, which was inconsistent with the sequencing results. This may be due to the small number of samples and the large individual differences. The results are shown in Figure 4 and Table 2.

### 3.5. CeRNA Interaction Network Analysis of lnc-ZNF32-1 : 1

In the lnc-ZNF32-1 : 1 ceRNA network map, the green polygon represents lnc-ZNF32-1 : 1, the red quadrilateral represents miRNA, and the pink oval represents mRNA. After the original data was corrected by background and standardized, 512 differentially expressed genes were obtained, of which 371 were upregulated and 141 were downregulated, as shown in Figure 5.

### 3.6. CeRNA Interaction Network Analysis of lnc-PCGF5-2 : 1

In the ceRNA network map of lnc-PCGF5-2 : 1, the green polygon represents lnc-PCGF5-2 : 1, the red quadrilateral represents miRNA, and the pink oval represents mRNA, see Figure 6.

### 3.7. lnc-ZNF32-1 : 1, lnc-PCGF5-2 : 1 Diagnostic Specificity, and Sensitivity Analysis

The results showed that lnc-ZNF32-1 : 1 (AUC = 0.7375, *P* = 0.01) and lnc-PCGF5-2 : 1 (AUC = 0.872, *P* < 0.0001) were highly specific and sensitive for diagnosis, which may be used as a standard for the diagnosis of ACI diseases. The results are shown in Figure 7.

## 4. Discussion

CI is a relatively common disease. Increasingly tight serious environment and unhealthy lifestyles lead to a trend of increasing CI in young people, which is a serious economic burden on the patients' family and society [22, 23]. Studies have found that in the acute phase of CI, many physiological and pathological processes are prone to occur, such as hypoxic-ischemic neurological disorders, excitatory amino acid neurotoxicity, calcium overload, programmed cell death or apoptosis, and microvascular disorder hypothesis. At the same time, there will be platelet coagulation abnormalities, stress blood pressure, and elevated blood glucose [8]. Due to the high incidence of CI and the complicated pathologies, it has been one of the hotspots of research in recent years.

In recent years, with the changes in medical models and the development of sequencing technology, research on various diseases has focused on noncoding and encoding genes, especially lncRNA. lncRNA is a relatively new type of RNA molecule that is greater than 200 nucleotides in length [24]. lncRNA has been reported to have a stable secondary structure, mainly exists in cytoplasm, and exhibits strong cell and tissue-specific expression [25]. In cardiovascular studies, lncRNA plays a crucial role in diseases such as atherosclerosis, heart failure, coronary heart disease, and myocardial infarction [26]. The expression profile of brain lncRNA has obvious changes in many pathological conditions, and lncRNA has far-reaching effects on the pathophysiological process of brain diseases [27–29]. Ng et al. [30] discussed a series of potential targets of lncRNAs and their promise as novel therapeutics and biomarkers in brain disorders. For example, lncRNA MALAT-1 was found upregulated in the cerebellum, hippocampus, and brain stem of the human alcoholic brain and following alcohol withdrawal in the rat [31]. During the occurrence and development of cerebral ischemia-reperfusion injury, lncRNA MALAT-1 downregulates miR-211-5p expression to promote neuronal damage by acting the expression of COX-2 [32]. Another well-known lncRNA linc-PINT plays neuroprotective role in Parkinson's disease [33]. In addition, genome-wide analysis identifies a novel linc-PINT splice variant associated with vascular amyloid pathology in Alzheimer's disease [34].

With the increasing research on the role of lncRNA in the human genome, researchers have found that complex networks regulated by lncRNA play an important role in cell and tissue differentiation. Cesana et al. [35] found that lncRNA can promote neuronal differentiation after interacting with transcription factors. Cao et al. [36] reported that lncRNA MD1 acts as a competing endogenous RNA that regulates muscle differentiation in mouse and human myoblasts. In recent years, researchers found that a large number of lncRNAs may play an important role in CI. Study has been proved that high expression of lncRNA MALAT-1 [37], MEG3 [38], MIAT [39], and GAS5 [40] exacerbates cerebral ischemia-reperfusion injury. In addition, lncRNA SNHG1 [41], NKILA [42], and ZFAS1 [43] functions as a protective factor in CI. However, there are few reports on lncRNA in clinical diagnosis of CI. In this study, we used lncRNA high-throughput to detect differential expression profiles of lncRNA and mRNA in patients with CI, to find specific lncRNA and mRNA and to introduce lncRNA and mRNA into the clinical target treatment of CI. Compared with the healthy group, there were 512 known differentially expressed lncRNAs in the serum of patients with CI, of which 371 were upregulated and 141 were downregulated; there were 421 known differentially expressed mRNAs, of which 245 were upregulated and 176 downregulated. In order to verify the reliability of high-throughput microarray detection, we randomly selected two lncRNAs with significant differences in expression and detected their expression levels by qRT-PCR. The expression of lnc-ZNF32-1 : 1 was significantly up-regulated in ACI group, which is consistent with the sequencing results. The expression of lnc-PCGF5-2 : 1 was significantly downregulated in the ACI group, which is contrary to the sequencing results, which may be due to the small number of sequencing samples and the large individual differences. A study [44] on lncRNA MIAT indicated that its expression level was significantly upregulated and correlated with National Institutes of Health Stroke Scale (NIHSS) scores and modified Rankin Scale and infarct volume in ischemic stroke patients, which means MIAT could serve as a potential marker for diagnosis of ischemic stroke. Ren et al. found that lncRNA UCA1 might sever as a candidate prognostic biomarker in acute ischemic stroke patients [45]. By contrast, our study lacks correlation analysis between lcnRNA expression level and patient treatment evaluation data.

Bioinformatics analysis was then performed, including GO analysis and KEGG pathway analysis to predict the functional roles of differential mRNA. GO analysis revealed that differentially expressed mRNA is enriched in multiple biological processes, which are related to neurodevelopment and cardiovascular and cerebrovascular diseases. The mRNA mainly interacts with organelles, supramolecular complexes, extracellular spaces, cell membranes, cell membrane lumens, extracellular regions, synapses, nuclei, signal sensors, molecular function regulators, transcriptional regulation, antioxidants, biological regulation, cell transformation, and cell proliferation. The KEGG pathway analysis showed that differentially upregulated mRNA genes are mainly involved in metabolic, endocrine-resistant pathways, cell carcinoma pathways, MAPK, mTOR, PI3K-AKT, and cellular multiplex pathways.

In summary, lncRNA is closely related to the occurrence, development, and repair of CI. lnc-ZNF32-1 : 1 and lnc-PCGF5-2 : 1 have high specificity and sensitivity for diagnosis and can be used as a standard for the diagnosis of ACI diseases. Although lnc-PCGF5-2 : 1 was downregulated in ACI group due to the insufficient amount of specimens in the verification process, the GO analysis, and KEGG pathway analysis was consistent with expectations. It is still necessary to carry out further verification experiments, as well as to investigate other differentially expressed lncRNAs for the optimal diagnosis of CI. In addition, to further understand lncRNA markers and their mechanisms in CI, the target genes and signal pathways that are closely related to lncRNA markers could be selected for further validations in the prospective experiments.

## Figures and Tables

**Figure 1:** Differential expression and cluster analysis of lncRNA expression in serum of ACI group and NC group. (a) Scatter plot of differentially expressed lncRNA. (b) Heat map of differentially expressed lncRNA.

**Figure 2:** Differential expression and cluster analysis of mRNA expression in serum of ACI group and NC group. (a) Scatter plot of differential genes. (b) Heat map of differential genes.

**Figure 3:** GO and KEGG analysis of differentially expressed genes in serum of ACI group and NC group. (a) GO analysis. (b) KEGG analysis.

**Figure 4:** Verification of differential expression of lncRNA in ACI and NC Groups. (a) Expression level of lnc-ZNF32-1 : 1 in serum. (b) Expression level of lnc-PCGF5-2 : 1 in serum (^∗^*P* < 0.05, ^∗∗∗^*P* < 0.001).

**Figure 5:** CeRNA interaction network analysis of lnc-ZNF32-1 : 1.

**Figure 6:** CeRNA interaction network analysis of lnc-PCGF5-2 : 1.

**Figure 7:** Diagnostic specificity and sensitivity analysis of lnc-ZNF32-1 : 1 and lnc-PCGF5-2 : 1 (lnc-ZNF32-1 : 1: AUC = 0.7375, *P* = 0.01; lnc-PCGF5-2 : 1: AUC = 0.872, *P* < 0.0001).

**Table 1:** Results of KEGG enrichment analysis of serum mRNA differentially expressed genes in ACI group and NC group.

Term	Input number	Background number	*P* value	Corrected *P* value
Endocrine resistance	7	97	0.000117037	0.022939175
Basal cell carcinoma	5	55	0.000419466	0.029101128
Pathways in cancer	13	397	0.000445425	0.029101128
HTLV-I infection	10	259	0.000600404	0.029419804
Melanogenesis	6	100	0.000902136	0.033794958
Signaling pathways regulating pluripotency of stem cells	7	142	0.00103454	0.033794958

**Table 2:** Select lnc-ZNF32-1 : 1 and lnc-PCGF5-2 : 1 for differentially expressed serum lncRNA in ACI group and NC group.

Table analyzed	Iinc-ZNF32-1 : 1	Inc-PCGF5-2:1
Column B	NC	NC
VS.	Vs.	Vs.
Column A	ACI	ACI
Unpaired *t* test		
*P* value	0.0232	0.0010
Significantly different? (*P* < 0.05)	Yes	Yes
One-or two-tailed *P* value?	Two-tailed	Two-tailed
*t*,df	*t* = 2.365 df-38	*t* = 3.538df = 42
How big is the difference?		
Mean t SEM of column A	2.396 ± 0.1818	0.7204 ± 0.1575
Mean t SEM of column B	1.525 ± 0.3200	3.367 ± 0.7644
Difference between means	−0.8705 ± 0.3680	2.647 ± 0.7480
95%6 confidence interval	-1.616 to-0.1255	1.137 to 4.156
*R* square	0.1283	0.2296.

## Data Availability

The data could be downloaded at (https://portal.gdc.cancer.gov/, and https://dcc.icgc.org/projects/LIRI-JP), and the code used in this study are available from the corresponding author on reasonable request.

## References

[1] Uchiyama S. (2006). Cerebral infarction. *Nihon Rinsho*.

[2] Saliou G., Théaudin M., Vincent C. J.-L., Souillard-Scemama R. (2014). General description of CI. *Practical Guide to Neurovascular Emergencies*.

[3] Titov B., Matveeva N., Martynov M. Y., Favorova O. O. (2015). Ischemic stroke as a complex polygenic disease. *Molecular Biology*.

[4] Tsai C.-F., Thomas B., Sudlow C. L. M. (2013). Epidemiology of stroke and its subtypes in Chinese vs white populations: a systematic review. *Neurology*.

[5] Liu H. (2011). Application of multimodal CT examination in acute cerebral infarction. *Guoji Naoxueguanbing Zazhi*.

[6] Spence J. D. (2018). Advances in stroke prevention. *Journal of International Translational Medicine*.

[7] Rigatelli G., Zuin M., Dell’Avvocata F., Nanjundappa A., Daggubati R., Nguyen T. (2018). Non-invasive evaluation of fluid dynamic of aortoiliac atherosclerotic disease: impact of bifurcation angle and different stent configurations. *Journal of International Translational Medicine*.

[8] Li M. T., Luo C. H., Xu P. J. (2018). Analysis of circRNA expression profile in patients with cerebral infarction. *Journal of Guangdong Medical College*.

[9] Sakamoto N., Honma R., Sekino Y. (2017). Non-coding RNAs are promising targets for stem cell-based cancer therapy. *Non-coding RNA Research*.

[10] Liang J., Chen W., Lin J. (2019). lncRNA: an all-rounder in rheumatoid arthritis. *Journal of Translational Internal Medicine*.

[11] Yang L., Froberg J. E., Lee J. T. (2014). Long noncoding RNAs: fresh perspectives into the RNA world. *Trends in Biochemical Sciences*.

[12] Asadi M. R., Hassani M., Kiani S. (2021). The perspective of dysregulated lncRNAs in Alzheimer's disease: a systematic scoping review. *Frontiers in Aging Neuroscience*.

[13] Wapinski O., Chang H. Y. (2011). Long noncoding RNAs and human disease. *Trends in Cell Biology*.

[14] Kataoka M., Wang D. Z. (2014). Non-coding RNAs including miRNAs and lncRNAs in cardiovascular biology and disease. *Cell*.

[15] Yamane S., Katada C., Tanabe S. (2017). Clinical outcomes in patients with cancer of unknown primary site treated by gastrointestinal oncologists. *Journal of Translational Internal Medicine*.

[16] Wang Y., Zhou Y., Hu Z. (2017). The functions of circulating tumor cells in early diagnosis and surveillance during cancer advancement. *Journal of Translational Internal Medicine*.

[17] Schizas D., Kapsampelis P., Mylonas K. S. (2018). Adenosquamous carcinoma of the esophagus: a literature review. *Journal of Translational Internal Medicine*.

[18] Michael J. S., Lee B. S., Zhang M., Yu J. S. (2018). Nanotechnology for treatment of glioblastoma multiforme. *Journal of Translational Internal Medicine*.

[19] Wilusz J. E., Sunwoo H., Spector D. L. (2009). Long noncoding RNAs: functional surprises from the RNA world. *Genes & Development*.

[20] Cabili M. N., Trapnell C., Goff L. (2011). Integrative annotation of human large intergenic noncoding RNAs reveals global properties and specific subclasses. *Genes & Development*.

[21] Neurology Professional Committee of Chinese Society of Integrated Traditional and Western Medicine (2018). Chinese guidelines for diagnosis and treatment of CI with integrated traditional Chinese and Western Medicine (2017). *Chinese Journal of Integrated Traditional and Western Medicine*.

[22] Neurology Professional Committee (2018). Chinese CI diagnosis and treatment guidelines by integrated Chinese and Western medicine (2017). *Chinese Journal of Integrated Traditional and Western Medicine*.

[23] Wang H., Cai H. (2015). The clinical curative effect observation of treating acute CI in the very early stage with acupuncture. *Journal of Clinical Acupuncture and Moxibustion*.

[24] Yang D., Liu Z., Luo Q. (2013). Plasma ghrelin and pro-inflammatory markers in patients with obstructive sleep apnea and stable coronary heart disease. *Medical Science Monitor*.

[25] Jiang Z. F., Zhang L. (2021). lncRNA: a potential research direction in intestinal barrier function. *Digestive Diseases and Sciences*.

[26] Graf J., Kretz M. (2020). From structure to function: route to understanding lncRNA mechanism. *BioEssays*.

[27] Yang S., Lim K. H., Kim S. H., Joo J. Y. (2021). Molecular landscape of long noncoding RNAs in brain disorders. *Molecular Psychiatry*.

[28] Yin K. J., Hamblin M., Chen Y. E. (2014). Non-coding RNAs in cerebral endothelial pathophysiology: emerging roles in stroke. *Neurochemistry International*.

[29] Dong X., Yu L. G., Sun R. (2013). Inhibition of PTEN expression and activity by angiotensin II induces proliferation and migration of vascular smooth muscle cells. *Journal of Cellular Biochemistry*.

[30] Ng S. Y., Johnson R., Stanton L. W. (2012). Human long non-coding RNAs promote pluripotency and neuronal differentiation by association with chromatin modifiers and transcription factors. *The EMBO Journal*.

[31] Kryger R., Fan L., Wilce P. A., Jaquet V. (2012). MALAT-1, a non protein-coding RNA is upregulated in the cerebellum, hippocampus and brain stem of human alcoholics. *Alcohol*.

[32] Tan X., Guo W., Peng Z. (2021). lncRNA-Malat1 down-regulates miR-211-5p expression to promote neuronal damage from cerebral ischemia reperfusion injury. *Biochemical Pharmacology*.

[33] Simchovitz A., Hanan M., Yayon N. (2020). A lncRNA survey finds increases in neuroprotective LINC-PINT in Parkinson’s disease substantia nigra. *Aging Cell*.

[34] Reddy J. S., Allen M., Ho C. C. G. (2021). Genome-wide analysis identifies a novel LINC-PINT splice variant associated with vascular amyloid pathology in Alzheimer's disease. *Acta Neuropathologica Communications*.

[35] Cesana M., Cacchiarelli D., Legnini I. (2011). A long noncoding RNA controls muscle differentiation by functioning as a competing endogenous RNA. *Cell*.

[36] Cao B., Liu N., Wang W. (2016). High glucose prevents osteogenic differentiation of mesenchymal stem cells via lncRNA AK028326/CXCL13 pathway. *Biomedicine & Pharmacotherapy*.

[37] Hu Y., Ye C., Cheng S., Chen J. (2021). Propofol downregulates lncRNA MALAT1 to alleviate cerebral ischemia-reperfusion injury. *Inflammation*.

[38] Liang J., Wang Q., Li J. Q., Guo T., Yu D. (2020). Long non-coding RNA MEG3 promotes cerebral ischemia-reperfusion injury through increasing pyroptosis by targeting miR-485/AIM2 axis. *Experimental Neurology*.

[39] Li S., Fu J., Wang Y., Hu C., Xu F. (2021). lncRNA MIAT enhances cerebral ischaemia/reperfusion injury in rat model via interacting with EGLN2 and reduces its ubiquitin-mediated degradation. *Journal of Cellular and Molecular Medicine*.

[40] Zhao J. H., Wang B., Wang X. H., Xu C. W. (2019). Effect of lncRNA GAS5 on the apoptosis of neurons via the notch1 signaling pathway in rats with cerebral infarction. *European Review for Medical and Pharmacological Sciences*.

[41] Chen J., Zhang W., Wu Y. Q., Chen H., Zhao J. F. (2019). lncRNA SNHG1 inhibits neuronal apoptosis in cerebral infarction rats through PI3K/Akt signaling pathway. *European Review for Medical and Pharmacological Sciences*.

[42] Gao W., Ning Y., Peng Y., Tang X., Zhong S., Zeng H. (2021). lncRNA NKILA relieves astrocyte inflammation and neuronal oxidative stress after cerebral ischemia/reperfusion by inhibiting the NF-*κ*B pathway. *Molecular Immunology*.

[43] Zhang Y., Zhang Y. (2020). lncRNA ZFAS1 improves neuronal injury and inhibits inflammation, oxidative stress, and apoptosis by sponging miR-582 and upregulating NOS3 expression in cerebral ischemia/reperfusion injury. *Inflammation*.

[44] Zhu M., Li N., Luo P. (2018). Peripheral blood leukocyte expression of lncRNA MIAT and its diagnostic and prognostic value in ischemic stroke. *Journal of Stroke and Cerebrovascular Diseases*.

[45] Ren B., Song Z., Chen L., Niu X., Feng Q. (2021). Long non-coding RNA UCA1 correlates with elevated disease severity, Th17 cell proportion, inflammatory cytokines, and worse prognosis in acute ischemic stroke patients. *Journal of Clinical Laboratory Analysis*.

